The article "Membrane fatty acid heterogeneity of leukocyte classes is altered during in vitro cultivation but can be restored with ad-hoc lipid supplementation" was published in 2015. Journal: Lipids Health Dis.

# Membrane fatty acid heterogeneity of leukocyte classes is altered during in vitro cultivation but can be restored with ad-hoc lipid supplementation

**DOI:** 10.1186/s12944-015-0166-3

**Published:** 2015-12-24

**Authors:** Paola Poggi, Roberto Mirabella, Simona Neri, Elisa Assirelli, Paolo Dolzani, Erminia Mariani, Philip C. Calder, Alexandros Chatgilialoglu

**Affiliations:** Remembrane Srl, via Selice 84/A, 40026 Imola, Italy; Laboratory of Immunorheumatology and Tissue Regeneration/RAMSES, Rizzoli Orthopedic Institute, via di Barbiano 1/10, 40136 Bologna, Italy; Department of Medical and Surgical Sciences, University of Bologna, Bologna, Italy; Human Development and Health Academic Unit, Faculty of Medicine, University of Southampton, Tremona Road, SO16 6YD Southampton, UK; NIHR Southampton Biomedical Research Centre, University Hospital Southampton NHS Foundation Trust and University of Southampton, Southampton, UK; Department of Biological Sciences, Faculty of Science, King Abdulaziz University, Jeddah, Saudi Arabia

**Keywords:** Leukocytes, Lymphocytes, Monocytes, Fatty acids, Lipid supplementation, Membrane fatty acid profile, Membrane lipid composition, Cell cultures

## Abstract

**Background:**

The cell membrane is a primary and fundamental player in most cellular processes, and fatty acids form a major structural component of cell membranes. The aim of this study was to compare the membrane fatty acid profiles of different human blood leukocytes and selected cell lines, to identify the effects of in vitro culture on fatty acid profiles, and to test medium supplements for their effect on fatty acid profiles.

**Methods:**

Different classes of leukocytes were isolated from human blood and their membrane fatty acid profiles were analysed and compared. After culturing in vitro immortalised and primary leukocytes, membrane fatty acids were analysed and compared. Finally, different lipid formulations were developed and used for supplementing leukocytes in vitro in an effort to maintain the in vivo fatty acid profile. Descriptive and analytical tests were performed to compare the obtained fatty acid profiles.

**Results:**

Membrane fatty acid profiles of primary human CD4^+^ T-lymphocytes, CD8^+^ T-lymphocytes, B-lymphocytes and monocytes differed. Moreover, there were differences among Jurkat, Raji and THP-1 cell lines and the corresponding primary leukocyte classes, as well as between freshly prepared and in vitro cultured primary lymphocytes. A lipid supplement was able to maintain cultured Jurkat cells with a membrane fatty acid profile almost identical to that of the primary CD4^+^ T-lymphocytes. Finally, variations in the lipid supplement composition enabled the development of Jurkat cells with different membrane fatty acid profiles characterising different physiological or pathological human conditions.

The article "Membrane fatty acid heterogeneity of leukocyte classes is altered during in vitro cultivation but can be restored with ad-hoc lipid supplementation" was published in 2015. Journal: Lipids Health Dis.

**Conclusions:**

Each leukocyte class has its own specific membrane fatty acid profile in vivo. Cultured primary leukocytes and immortalized leukocytic cells display different membrane fatty acid profiles when compared to their respective in vivo counterparts. The membrane fatty acid composition of cultured cells can be restored to reflect that of the corresponding in vivo condition through use of optimised lipid supplementation. Typical physiological or pathological leukocyte membrane fatty acid profiles can be obtained by tuning in vitro fatty acid supplementation.

## Background

The plasma membrane of cells provides a physical barrier separating the contents of a cell from its surroundings, but allowing for specific communication with the extracellular environment through receptors, transporters and so on and for the generation of intracellular signals that are key to cellular responsiveness. The lipid composition of the plasma membrane has long been recognized to be important in creating the environment in which membrane proteins can function [1] and in providing the substrates from which many second messengers are generated [2]. More recent studies have identified membrane lipid rafts as vital functional components of cellular responses [3–5] and membrane lipids as being responsible for coordinating many core aspects of cell metabolism [6–8]. Among the many lipid species characterising cell membranes, fatty acids are the predominant structural component and can constitute up to 80 % in weight of the lipid part of the membrane. Cell membrane fatty acids are typically 14 to 24 carbons in length and contain between 0 and 6 double bonds, these structural characteristics strongly influencing the biophysical and functional properties of the membrane [9, 10]. Taken individually or in bulk, membrane fatty acids influence fundamental properties of the cell, such as membrane fluidity [6, 11], protein folding and functionality [12], lipid rafts and signalling [13–15], and trafficking processes [16, 17], among others. As an example, many of the functional effects of fatty acids on inflammation and immunity relate to the incorporation of the fatty acids into the membranes of the cells involved in those processes from where they exert their effects [18, 19].

The function of cells is often examined in culture systems using either primary cells isolated from humans or experimental animals or using immortalised cell lines. Despite the widespread use of cell cultures, this approach suffers from high variability and technical limitations, perhaps made worse by the use of animal-derived components and non-standardised sera. Even the impressive recent technological advances, such as 3D cultures and Body-on-Chips, do not allow current models to be completely reliable, with many variables still not considered. At present, cell culture technology is far from being a completely predictable experimental model able to reproduce in vivo cell physiology and behaviour; this variance leads to scientific data and pre-clinical studies which often are unreliable and misleading. In particular, despite its proven importance, membrane lipid content, composition and behaviour are poorly considered during cell culture. Furthermore, due to significant alterations of the fatty acid content and composition of the cell membrane, and consequently also of its biophysical and functional properties, during culture cells differ greatly from their corresponding in vivo comparators [20, 21]. This introduces substantial biases in most in vitro studies, with serious consequences for the reliability of experimental data, weakening the usefulness of in vitro research and resulting in significant waste of time and resources.

The article "Membrane fatty acid heterogeneity of leukocyte classes is altered during in vitro cultivation but can be restored with ad-hoc lipid supplementation" was published in 2015. Journal: Lipids Health Dis.

The fatty acid composition of leukocytes has been widely reported and linked to the ability of specific fatty acids to influence immune and inflammatory responses [19, 22–24]. In fact, leukocytes have a specific fatty acid profile, which differs amongst different leukocyte classes and is finely tuned in time and space for their specific functions [25–27]. In addition, the fatty acid composition of the leukocyte membrane is subject to significant variations deriving from individual dietary habits [28]. These aspects are not taken into account in current cell culture approaches, and this causes in vitro studies to be often unreliable and misleading.

The objective of the current study was to expand our knowledge of membrane fatty acid composition of primary human leukocyte classes, the influence of cell culture on such composition, and how primary leukocytes compare with immortalised leukocyte-derived cell lines. To our knowledge, this is the first study addressing this intriguing issue. Our pre-study hypothesis was that cultured leukocytes will differ in membrane fatty acid composition from the corresponding primary leukocytes, thus highlighting the importance of a correct ad-hoc in vitro supplementation to create culture conditions to maintain or reinstate fatty acid composition seen in vivo.

## Methods

### Study population

Peripheral blood mononuclear cells (PBMCs) were obtained from buffy coat preparations derived from the whole blood of 8 healthy male donors anonymously identified by code numbers (mean age 48.5 ± 13.4 years). Buffy coats no more available for clinical use (not used within 24 h after collection) were provided by the Transfusion Unit of the Ospedale Maggiore (Bologna) as approved by the Centro Regionale Sangue (Prot. N.32041/10-14-01).

The article "Membrane fatty acid heterogeneity of leukocyte classes is altered during in vitro cultivation but can be restored with ad-hoc lipid supplementation" was published in 2015. Journal: Lipids Health Dis.

### Mononuclear cell isolation and CD14^+^, CD8^+^, CD19^+^ and CD4^+^ cell purification

PBMCs were isolated by conventional density gradient centrifugation over Lympholyte-H gradient medium (*ρ* = 1.077 ± 0.001 g/cm^3^; Cedarlane, USA). Briefly, buffy coats were diluted with 3 volumes of PBS and layered over Lympholyte-H (at a 2:1 ratio) in 50 ml conical tubes, then centrifuged at 800 × g for 20 min at room temperature. PBMCs collected at the interphase were washed twice with PBS (400 × g for 10 min), counted and resuspended in PBS containing 0.5 % fatty acid-free bovine serum albumin (GE Healthcare, Milan, Italy) and 2 mM EDTA, pH 8.0. PBMCs were then immediately used for purification of cellular subpopulations.

CD14^+^, CD19^+^ and CD8^+^ cellular subpopulations were purified using an AutoMACS Pro Separator (Miltenyi Biotec, Bologna, Italy) and specific microbeads for positive selection (CD14, CD19 and CD8 Microbeads; Miltenyi Biotec, Bologna, Italy). The CD4^+^ cell population was positively purified from the CD14 negative eluted fraction with the same instrument and CD4 Microbeads (Miltenyi Biotec, Bologna, Italy). MACS isolated cell subsets were collected, counted and an aliquot of those subsets was used to assess population purity. Cells were incubated for 15 min at room temperature with FITC-conjugated antibodies against CD14, CD19, CD8 and CD4 (Miltenyi Biotec, Bologna, Italy), washed twice in PBS and evaluated by flow cytometry (FACSCanto II, BD). FITC fluorescence was filtered by a 530 ± 21 bandpass filter. The frequency of positive cells was measured as the percentage of gated cells in the FITC channel with activities above 99 % of the corresponding isotype control. Purities of the obtained cell populations were (mean ± SD): 91.9 ± 3.7 % for CD14^+^, 93.8 ± 6.9 % for CD19^+^, 92.4 ± 4.4 % for CD8^+^ and 94.9 ± 3.7 % for CD4^+^. Freshly isolated cell populations were washed, lysed and pelleted as described below.

### In vitro cultures

All cell culture media, sera and reagents were purchased from Euroclone SpA, Milan, Italy. Immortalised leukocytic cell lines (Jurkat, Raji and THP-1 cells) were kindly provided by Rizzoli Orthopedic Institute and University of Bologna. Jurkat, Raji and THP-1 cells were cultured in RPMI-1640 medium containing 10 % fetal bovine serum (FBS), L-glutamine (2 mM), penicillin (100 U/ml), and streptomycin (100 μg/ml). Cells were maintained in a humidified environment at 37 °C and 5 % CO_2_ and cultured in polystyrene culture flasks. Cells were passaged every 3 days, thus maintaining cell number between 1 × 10^5^ and 1 × 10^6^ per ml of medium (Jurkat cells), between 4 × 10^5^ and 3 × 10^6^ per ml of medium (Raji cells), or between 2 × 10^5^ and 1 × 10^6^ per ml of medium (THP-1 cells), according to the standard protocol provided by the American Type Culture Collection (ATCC).

The article "Membrane fatty acid heterogeneity of leukocyte classes is altered during in vitro cultivation but can be restored with ad-hoc lipid supplementation" was published in 2015. Journal: Lipids Health Dis.

To compare freshly isolated healthy human lymphocytes with primary cultured lymphocytes, PBMCs were isolated from the buffy coat of a 40 year old healthy male donor on a density gradient, as described above. Cells recovered from the gradient interphase were washed in PBS, resuspended in RPMI supplemented with 10 % FBS, counted and seeded in flasks at a density of 2 × 10^6^ cells/ml for 3 h to allow monocyte adherence. After this time, lymphocytes were recovered and maintained in culture in RPMI-1640 medium supplemented with 10 % FBS for 96 h in the absence or presence of 20 μg/ml phytohaemagglutinin (PHA) and then recovered. Freshly isolated and 96-h cultured lymphocytes were washed, lysed and pelleted as described below.

### Membrane isolation

Cells (7 × 10^6^) were collected in a 15 ml tube, centrifuged at 500 × *g* for 5 min and resuspended in 10 ml of PBS. The wash was repeated five times in order to discard traces of medium and serum used during the culture process. Cells were then resuspended into 500 μl of PBS and collected in a 1 ml tube, to which 500 μl of sterile H_2_O were added. Cells were then centrifuged for 30 min at 15,000 × *g* in a refrigerated centrifuge at 4 °C. The collected membranes were resuspended in 1 ml of PBS:H_2_O 1:1 and washed 5 times following the same procedure.

### Fatty acid composition analysis

Cell and cell membrane lipids were extracted with CHCl_3_/MeOH 2:1 (vol/vol) and then incubated with 0.5 M KOH in methanol for 10 min at room temperature, thus trans-esterifying fatty acids linked by ester bonds to alcohols. The corresponding fatty acid methyl esters (FAMEs) were formed, extracted with n-hexane and separated by gas chromatography. FAMEs were separated by gas-chromatography in an Agilent 7820A GC System (Agilent Technologies, Santa Clara, USA) fitted with a 30 m × 0.32 mm DB23 capillary column, film thickness 0.25 μm, and a Flame Ionization Detector (FID). Helium was used as carrier gas at 2.54 ml/min and the spilt injector was used with a split ratio of 10:1. Injector temperature was 250 °C and detector temperature was 260 °C. The column oven temperature was maintained at 50 °C for 2 min after sample injection and was programmed for the following temperature gradient: 10 °C/min from 50 °C to 180 °C, 3 °C/min from 180 °C to 200 °C and holding at 200 °C for 6 min. The separation was recorded with G6714AA SW EZChrom Elite Compact (Agilent Technologies). FAMEs were identified by comparison with standards purchased from NuCheckPrep Inc., Elysian, USA. FAMEs are expressed in weight %, based upon the % contribution of the peak area of each FAME in the chromatogram. To take into account the different signal of the detector for different molecules, a correction factor was applied to the experimental data coming from the integration of the chromatograms. The total of the peaks analysed for each chromatographic run was 100.

The article "Membrane fatty acid heterogeneity of leukocyte classes is altered during in vitro cultivation but can be restored with ad-hoc lipid supplementation" was published in 2015. Journal: Lipids Health Dis.

Fatty acid aggregates were calculated as follows:

Ʃ SFA = 14:0 + 15:0 + 16:0 + 17:0 + 18:0 + 20:0 + 22:0 + 23:0 + 24:0;

Ʃ MUFA = 16:1n-7 + 18:1n-9 + 18:1n-7 + 20:1n-9 + 22:1n-9 + 24:1n-9;

Ʃ PUFA = 18:2n-6 + 18:3n-6 + 18:3n-3 + 20:3n-9 + 20:3n-6 + 20:4n-6 + 20:3n-3 + 20:5n-3 + 22:2n-6 + 22:4n-6 + 22:5n-6 + 22:5n-3 + 22:6n-3;

Ʃ trans FA = t16:1n-7 + t18:1n-9;

Ʃ Omega3 = 18:3n-3 + 20:3n-3 + 20:5n-3 + 22:5n-3 + 22:6n-3;

Ʃ Omega6 = 18:2n-6 + 18:3n-6 + 20:3n-6 + 20:4n-6 + 22:2n-6 + 22:4n-6 + 22:5n-6;

Ʃ Omega7 = 16:1n-7 + 18:1n-7;

Ʃ Omega9 = 18:1n-9 + 20:1n-9 + 22:1n-9 + 24:1n-9.

Indexes were calculated as follows:

Unsaturation Index (UI) = Ʃ [mi*ni], where mi = mole percentage, ni = n° of double bonds;

Peroxidability Index (PI) = Ʃ monoenoic*0.025 + Ʃ dienoic + Ʃ trienoic*2 + Ʃ tetraenoic*3 + Ʃ pentaenoic*6 + Ʃ hexaenoic*8.

### Refeed® supplements

Refeed® supplements (Remembrane Srl, Imola, Italy) are a completely defined combination of non-animal derived lipids and antioxidants (NuCheckPrep Inc., Elysian, USA; Sigma Aldrich, St. Louis, USA; Applichem an ITW Inc., Chicago, USA) solubilised in 1 ml of ethanol (Sigma Aldrich). 1 ml of Refeed® was diluted in 560 ml of complete cell growth medium, the resulting ethanol concentration being < 1 % (vol/vol) in the final medium. Refeed® WT (Wild-Type), Refeed® CVD (Cardiovascular Disease) and Refeed® O3+ (Omega-3 plus) were specifically developed for Jurkat cells and their compositions are shown in Table 1.

**Table 1:** Composition of supplements used in the study

	Refeed WT	Refeed CVD	Refeed O3+
Lipids	19.50	19.00	18.10
Antioxidants	5.35	0.48	7.48

Composition of Refeed® WT, Refeed® CVD, Refeed® O3+ used for in-vitro supplementation of Jurkat cells. Data are the amount (mg) per 561 ml of complete medium

### Statistical analysis

Descriptive and analytical tests were performed with IBM SPSS® Statistics, Version 21.0. Data were checked for normality using the Shapiro-Wilk normality test. Normally distributed data were compared using Student’s *t*-test, to determine if two sets of fatty acid data were significantly different from each other. Non-normally distributed data were compared using the Mann–Whitney *U*-test. For sums and other aggregates (UI, PI), Student's *t*-test was performed when the aggregate was composed of all normally distributed individual FAMEs, while Mann–Whitney *U*-test was performed when the aggregate was composed of one or more not normally distributed FAMEs. For each test, the significance threshold was *P* < 0.05.

The article "Membrane fatty acid heterogeneity of leukocyte classes is altered during in vitro cultivation but can be restored with ad-hoc lipid supplementation" was published in 2015. Journal: Lipids Health Dis.

## Results

### Primary leukocyte classes have different membrane fatty acid compositions from one another

From the blood of 8 healthy individuals, four categories of leukocytes were isolated: CD4^+^ T-lymphocytes (helper T cells), CD8^+^ T-lymphocytes (cytotoxic T cells), CD19^+^ (B-lymphocytes) and CD14^+^ (monocytes). Their membrane fatty acid compositions are reported in Table 2. Data show a number of significant differences among leukocyte classes, spread among individual fatty acids, fatty acid sums and indexes. The five most prevalent fatty acids in all four cell types were palmitic (16:0), stearic (18:0), arachidonic (20:4n-6), oleic (18:1n-9) and linoleic (18:2n-6), typically in that order. Among those five fatty acids monocytes had the lowest proportions of palmitic and stearic and the highest proportions of oleic and arachidonic (Table 2). Docosahexaenoic acid (22:6n-3) was present in all cell types at about 2 to 3 % by weight of total fatty acids (Table 2). As a result of the differences in individual fatty acids, the sum of fatty acids of different classes differed among the cell types (Table 2). In particular monocytes had a lower proportion of saturated fatty acids and higher proportions of monounsaturated fatty acids, PUFAs and n-6 PUFAs (Table 2). Furthermore monocytes had higher UI and PI, reflecting the higher PUFA content (Table 2). The total n-6 to n-3 PUFA ratio among the different cell types was around 5.

**Table 2:** Membrane fatty acid profiles of primary human leukocytes

	CD4+	CD8+	CD19+	CD14+
14:0	0,635 ± 0,190^abc^	0,869 ± 0,185^ae^	0,923 ± 0,215^bf^	0,413 ± 0,157^cef^
15:0	0,256 ± 0,150^abc^	0,412 ± 0,125^ae^	0,430 ± 0,139^bf^	0,180 ± 0,107^cef^
16:0	27,156 ± 1,864^abc^	29,451 ± 2,352^ade^	31,780 ± 3,523^bdf^	20,373 ± 2,321^cef^
t16:1n-7	0,265 ± 0,133	0,364 ± 0,156	0,397 ± 0,171	0,203 ± 0,097
16:1n-7	0,257 ± 0,140	0,341 ± 0,161	0,358 ± 0,174	0,255 ± 0,080
17:0	0,696 ± 0,169^c^	0,922 ± 0,258^e^	0,879 ± 0,210^f^	0,435 ± 0,067^cef^
18:0	26,877 ± 3,827	28,296 ± 3,344^e^	30,470 ± 4,447^f^	24,146 ± 2,354^ef^
t18:1n-9	0,012 ± 0,033	0,021 ± 0,060	0,020 ± 0,057	0,039 ± 0,063
18:1n-9	7,919 ± 1,053^abc^	6,383 ± 1,044^ae^	7,083 ± 3,024^bf^	14,440 ± 1,039^cef^
18:1n-7	2,208 ± 0,375^abc^	1,662 ± 0,424^a^	1,431 ± 0,199^b^	1,552 ± 0,225^c^
18:2n-6	6,946 ± 1,323^ab^	5,071 ± 0,803^ae^	4,705 ± 0,878^bf^	6,577 ± 0,772^ef^
18:3n-6	0,179 ± 0,118	0,229 ± 0,138	0,206 ± 0,183	0,167 ± 0,091
18:3n-3	0,396 ± 0,319	0,601 ± 0,232^e^	0,536 ± 0,280^f^	0,180 ± 0,090^ef^
20:0	0,697 ± 0,241^ab^	1,096 ± 0,241^ae^	1,156 ± 0,215^bf^	0,533 ± 0,109^ef^
20:1n-9	0,806 ± 0,475	1,141 ± 0,995	0,896 ± 0,846	0,672 ± 0,249
20:3n-9	0,765 ± 0,090^abc^	0,513 ± 0,116^a^	0,608 ± 0,132^b^	0,618 ± 0,087^c^
20:3n-6	1,519 ± 0,396^b^	1,009 ± 0,332	0,899 ± 0,318^bf^	1,357 ± 0,304^f^
20:4n-6	12,755 ± 2,656^bc^	9,251 ± 3,097^e^	8,240 ± 4,173^bf^	16,422 ± 2,357^cef^
20:3n-3	0,041 ± 0,076	0,059 ± 0,119	0,000 ± 0,000	0,025 ± 0,059
20:5n-3	0,098 ± 0,112	0,166 ± 0,301	0,113 ± 0,165	0,138 ± 0,100
22:0	0,978 ± 0,579^abc^	1,642 ± 0,591^ae^	1,356 ± 0,435^bf^	0,492 ± 0,152^cef^
22:1n-9	1,588 ± 0,595	2,725 ± 1,570^e^	2,014 ± 1,418^f^	0,664 ± 0,430^cef^
22:2n-6	0,000 ± 0,000	0,024 ± 0,067	0,000 ± 0,000	0,031 ± 0,045
23:0	0,216 ± 0,277	0,239 ± 0,250	0,087 ± 0,175	0,057 ± 0,053
22:4n-6	1,816 ± 0,314^c^	2,662 ± 1,945^e^	1,545 ± 0,610^f^	3,553 ± 0,446^cef^
22:5n-6	0,356 ± 0,110^c^	0,234 ± 0,189^e^	0,431 ± 0,754	0,624 ± 0,227^ce^
22:5n-3	1,300 ± 0,444^abc^	0,855 ± 0,315^ae^	0,726 ± 0,279^bf^	2,376 ± 0,445^cef^
24:0	0,557 ± 0,345	0,809 ± 0,737^e^	0,606 ± 0,292	0,307 ± 0,135^e^
22:6n-3	2,672 ± 1,315	2,852 ± 2,253	2,040 ± 1,799	3,050 ± 1,187
24:1n-9	0,035 ± 0,098	0,098 ± 0,276	0,064 ± 0,180	0,123 ± 0,149
Ʃ SFA	58,067 ± 5,419^bc^	63,738 ± 5,544^e^	67,687 ± 7,719^bf^	46,936 ± 4,789^cef^
Ʃ MUFA	12,812 ± 1,675c	12,351 ± 2,609^e^	11,846 ± 3,172^f^	17,705 ± 1,311^cef^
Ʃ PUFA	28,844 ± 4,890^bc^	23,526 ± 4,114^de^	20,049 ± 5,101^bdf^	35,118 ± 3,867^cef^
Ʃ trans FA	0,276 ± 0,125	0,385 ± 0,135	0,417 ± 0,172	0,241 ± 0,100
Ʃ Omega3	4,507 ± 1,587	4,533 ± 2,154	3,415 ± 1,870^f^	5,770 ± 1,552^f^
Ʃ Omega6	23,572 ± 4,204^b^	18,481 ± 4,052^e^	16,026 ± 5,418^bf^	28,730 ± 3,304^ef^
Ʃ Omega7	2,465 ± 0,376bc	2,004 ± 0,477	1,789 ± 0,313^b^	1,806 ± 0,291^c^
Ʃ Omega9	11,112 ± 1,515^c^	10,861 ± 2,450^e^	10,665 ± 3,083^f^	16,516 ± 1,116^cef^
UI	109,691 ± 17,760^bc^	92,754 ± 17,734^e^	78,864 ± 20,728^bf^	141,417 ± 15,994^cef^
PI	91,565 ± 17,034^c^	79,091 ± 19,319^e^	65,462 ± 16,533^f^	118,882 ± 15,487^cef^

Membrane fatty acid profiles of different populations of primary human leukocytes (CD4^+^, CD8^+^, CD14^+^, CD19^+^). Data are expressed as mean (± SD) weight % of total membrane fatty acids (*n* = 8). ^a, b, c, d, e, f^ Statistically significant difference (*P* < 0.05) as follows: ^a^ CD4^+^ vs CD8^+^, ^b^ CD4^+^ vs CD19^+^, ^c^ CD4^+^ vs CD14^+^, ^d^ CD8^+^ vs CD19^+^, ^e^ CD8^+^ vs CD14^+^, ^f^ CD19^+^ vs CD14^+^

The article "Membrane fatty acid heterogeneity of leukocyte classes is altered during in vitro cultivation but can be restored with ad-hoc lipid supplementation" was published in 2015. Journal: Lipids Health Dis.

### Immortalised leukocyte cell lines have different membrane fatty acid compositions from one another

Three of the most common leukocytic cell lines used in research, corresponding to the categories of leukocytes described in Table 2, were selected for study. Jurkat (T-lymphocytes), Raji (B-lymphocytes), THP-1 (monocytes) cells were cultivated in vitro following the standard protocol provided by ATCC. The fatty acid compositions of these cells are shown in Table 3. Membrane fatty acid profiles were rather homogeneous among the three immortalised cell lines, being characterised by significant proportions of palmitic, stearic and oleic acids and rather low proportions of PUFAs, in particular of n-6 PUFAs, and especially of arachidonic acid (Table 3). The proportions of palmitoleic acid (16:1n-7) and 18:1n-7 were high (Table 3). Overall, these cell lines displayed low values for UI and PI.

**Table 3:** Membrane fatty acid profiles of Jurkat, Raji and THP-1 cell lines

	Jurkat	Raji	THP-1
9:0	0,000 ± 0,000	0,046 ± 0,046	0,028 ± 0,062
12:0	0,056 ± 0,011	0,052 ± 0,015	0,062 ± 0,013
14:0	2,062 ± 0,085^ab^	1,647 ± 0,093^ac^	2,876 ± 0,064^bc^
14:1n-5	0,047 ± 0,028	0,000 ± 0,000^c^	0,062 ± 0,006^c^
15:0	0,194 ± 0,012^ab^	0,526 ± 0,074^ac^	0,332 ± 0,013^bc^
16:0	25,776 ± 2,014^b^	23,959 ± 1,124^c^	28,740 ± 0,998^bc^
t16:1n-7	0,834 ± 0,036^ab^	1,345 ± 0,108^ac^	2,138 ± 0,022^bc^
16:1n-7	7,188 ± 0,407^ab^	1,656 ± 0,085^ac^	5,331 ± 0,221^bc^
17:0	0,411 ± 0,050^a^	0,679 ± 0,071^ac^	0,452 ± 0,013^c^
17:1n-7	0,000 ± 0,000^ab^	0,695 ± 0,05^ac^	0,410 ± 0,014^bc^
18:0	18,049 ± 0,606^ab^	20,329 ± 0,837^ac^	16,379 ± 1,056^bc^
t18:1n-9	0,735 ± 0,033^ab^	0,000 ± 0,000^a^	0,000 ± 0,000^b^
18:1n-9	24,938 ± 1,156^ab^	20,063 ± 0,945^a^	22,013 ± 0,585^b^
18:1n-7	5,521 ± 0,356^ab^	8,007 ± 0,437^ac^	6,932 ± 0,205^bc^
18:2n-6	3,144 ± 0,210^ab^	3,893 ± 0,115^ac^	1,499 ± 0,053^bc^
18:3n-6	0,094 ± 0,017^ab^	0,045 ± 0,013^a^	0,042 ± 0,007^b^
18:3n-3	0,302 ± 0,036^b^	0,324 ± 0,05^c^	0,124 ± 0,017^bc^
20:0	0,608 ± 0,045^ab^	0,421 ± 0,037^ac^	0,476 ± 0,014^bc^
20:1n-9	0,942 ± 0,091^ab^	2,334 ± 0,091^ac^	0,469 ± 0,010^bc^
20:3n-9	0,302 ± 0,012^ab^	0,635 ± 0,066^ac^	1,005 ± 0,039^bc^
20:3n-6	0,108 ± 0,007^ab^	1,222 ± 0,042^ac^	0,983 ± 0,069^bc^
20:4n-6	2,166 ± 0,109^ab^	4,347 ± 0,511^ac^	3,501 ± 0,122^bc^
20:3n-3	0,000 ± 0,000^ab^	0,097 ± 0,013^a^	0,094 ± 0,006^b^
20:5n-3	0,042 ± 0,013^ab^	0,572 ± 0,038^ac^	0,509 ± 0,018^bc^
22:0	0,946 ± 0,114^ab^	0,409 ± 0,018^ac^	0,455 ± 0,034^bc^
22:1n-9	0,144 ± 0,018^ab^	0,223 ± 0,024^ac^	0,052 ± 0,006^bc^
22:2n-6	0,000 ± 0,000^ab^	0,117 ± 0,018^ac^	0,077 ± 0,005^bc^
23:0	0,056 ± 0,013	0,089 ± 0,015^c^	0,040 ± 0,007^c^
22:4n-6	0,747 ± 0,103^b^	0,684 ± 0,092^c^	0,231 ± 0,031^bc^
22:5n-6	0,164 ± 0,026^b^	0,216 ± 0,034	0,252 ± 0,020^b^
22:5n-3	1,074 ± 0,121^ab^	1,723 ± 0,069^ac^	1,364 ± 0,038^bc^
24:0	0,000 ± 0,000^a^	0,073 ± 0,026^ac^	0,000 ± 0,000^c^
22:6n-3	1,479 ± 0,077^ab^	2,835 ± 0,093^a^	2,915 ± 0,117^b^
24:1n-9	1,872 ± 0,190^ab^	0,737 ± 0,071^ac^	0,160 ± 0,024^bc^
Ʃ SFA	48,158 ± 1,776	48,229 ± 1,23	49,839 ± 1,498
Ʃ MUFA	40,653 ± 1,636^ab^	33,715 ± 1,303^a^	35,429 ± 1,032^b^
Ʃ PUFA	9,621 ± 0,343^ab^	16,711 ± 0,464^ac^	12,594 ± 0,465^bc^
Ʃ trans FA	1,569 ± 0,034^ab^	1,345 ± 0,108^ac^	2,138 ± 0,022^bc^
Ʃ Omega3	2,896 ± 0,153^ab^	5,552 ± 0,145^ac^	5,006 ± 0,157^bc^
Ʃ Omega5	0,047 ± 0,028	0,000 ± 0,000^c^	0,062 ± 0,006^c^
Ʃ Omega6	6,422 ± 0,208^a^	10,525 ± 0,555^ac^	6,584 ± 0,271^c^
Ʃ Omega7	12,709 ± 0,509^a^	10,358 ± 0,511^ac^	12,673 ± 0,435^c^
Ʃ Omega9	28,199 ± 1,160^ab^	23,992 ± 0,959^a^	23,698 ± 0,648^b^
UI	73,097 ± 2,362^ab^	92,332 ± 1,687^ac^	83,240 ± 2,764^bc^
PI	43,162 ± 1,357^ab^	69,931 ± 1,054^ac^	62,191 ± 2,232^bc^

Data are expressed as mean (± SD) weight % of total membrane fatty acids (*n* = 5). ^a, b, c^ Statistically significant difference (*P* < 0.05) as follows: ^a^ Jurkat vs Raji, ^b^ Jurkat vs THP-1, ^c^ Raji vs THP-1

The article "Membrane fatty acid heterogeneity of leukocyte classes is altered during in vitro cultivation but can be restored with ad-hoc lipid supplementation" was published in 2015. Journal: Lipids Health Dis.

### Primary leukocyte classes have different membrane fatty acid compositions from their corresponding immortalised cell lines

Table 4 compares the fatty acid compositions of primary human leukocytes and their corresponding immortalised cell lines; these data are the same as those shown in Tables 2 and 3. The comparisons are: CD4^+^ and CD8^+^ T lymphocytes against Jurkat, CD19^+^ against Raji, and CD14^+^ against THP-1. These data clearly demonstrate that significant differences exist between the membrane fatty acid profiles of in vitro cell lines and those of the corresponding primary leukocytes, considering both individual fatty acids and fatty acid sums and indexes. Palmitic acid was higher in B lymphocytes (CD19^+^ cells) than in Raji cells and was lower in monocytes (CD14^+^ cells) than THP-1 cells. The cell lines had much higher proportions of palmitoleic acid, 18:1n-7 and oleic acid than primary human leukocytes. Conversely, the cell lines had lower proportions of stearic, linoleic and arachidonic acids. Interestingly docosahexaenoic acid was fairly similar between cell lines and primary leukocytes. Overall the cell lines had lower proportions of saturated fatty acids and especially PUFAs, particularly n-6 PUFAs, and higher proportions of monounsaturated fatty acids (Table 4). Consequently UI and PI values were lower for cell lines compared with primary leukocytes.

**Table 4:** Comparison of membrane fatty acid profiles between immortalised cell lines and corresponding primary leukocyte classes

	Jurkat	CD4+	CD8+	Raji	CD19+	THP1	CD14+
9:0	0,000 ± 0,000	0,000 ± 0,000	0,000 ± 0,000	0,046 ± 0,046	0,000 ± 0,000	0,000 ± 0,000	0,000 ± 0,000
12:0	0,056 ± 0,011	0,000 ± 0,000*	0,000 ± 0,000*	0,052 ± 0,015	0,000 ± 0,000*	0,041 ± 0,025	0,000 ± 0,000*
14:0	2,062 ± 0,085	0,635 ± 0,190*	0,870 ± 0,185*	1,647 ± 0,093	0,923 ± 0,215*	2,313 ± 0,493	0,413 ± 0,157*
14:1n-5	0,047 ± 0,028	0,000 ± 0,000*	0,000 ± 0,000*	0,000 ± 0,000	0,000 ± 0,000	0,041 ± 0,009	0,000 ± 0,000*
15:0	0,194 ± 0,012	0,256 ± 0,150*	0,412 ± 0,125*	0,526 ± 0,074	0,430 ± 0,139	0,324 ± 0,017	0,180 ± 0,107*
16:0	25,776 ± 2,014	27,156 ± 1,864	29,451 ± 2,352*	23,959 ± 1,124	31,780 ± 3,523*	28,591 ± 0,655	20,373 ± 2,321*
t16:1n-7	0,834 ± 0,036	0,265 ± 0,133*	0,364 ± 0,156*	1,345 ± 0,108	0,397 ± 0,171*	1,766 ± 0,074	0,203 ± 0,097*
16:1n-7	7,188 ± 0,407	0,257 ± 0,140*	0,341 ± 0,161*	1,656 ± 0,085	0,358 ± 0,174*	4,177 ± 0,195	0,255 ± 0,080*
17:0	0,411 ± 0,050	0,696 ± 0,169*	0,922 ± 0,258*	0,679 ± 0,071	0,879 ± 0,210	0,458 ± 0,076	0,435 ± 0,067
17:1n-7	0,000 ± 0,000	0,000 ± 0,000	0,000 ± 0,000	0,695 ± 0,050	0,000 ± 0,000*	0,436 ± 0,004	0,000 ± 0,000*
18:0	18,049 ± 0,606	26,877 ± 3,827*	28,296 ± 3,344*	20,329 ± 0,837	30,470 ± 4,447*	14,511 ± 0,640	24,146 ± 2,354*
t18:1n-9	0,735 ± 0,033	0,012 ± 0,033*	0,021 ± 0,060*	0,000 ± 0,000	0,020 ± 0,057	0,000 ± 0,000	0,039 ± 0,063
18:1n-9	24,938 ± 1,156	7,919 ± 1,053*	6,383 ± 1,044*	20,063 ± 0,945	7,083 ± 3,024*	22,967 ± 0,300	14,440 ± 1,039*
18:1n-7	5,521 ± 0,356	2,208 ± 0,375*	1,662 ± 0,424*	8,007 ± 0,437	1,431 ± 0,199*	7,906 ± 0,072	1,552 ± 0,225*
18:2n-6	3,144 ± 0,210	6,946 ± 1,323*	5,071 ± 0,803*	3,893 ± 0,115	4,705 ± 0,878	1,626 ± 0,161	6,577 ± 0,772*
18:3n-6	0,094 ± 0,017	0,179 ± 0,118	0,229 ± 0,138	0,045 ± 0,013	0,206 ± 0,183	0,037 ± 0,007	0,167 ± 0,091*
18:3n-3	0,302 ± 0,036	0,396 ± 0,319	0,601 ± 0,232*	0,324 ± 0,050	0,536 ± 0,280	0,130 ± 0,009	0,180 ± 0,090
20:0	0,608 ± 0,045	0,697 ± 0,241	1,096 ± 0,241*	0,421 ± 0,037	1,156 ± 0,215*	0,406 ± 0,026	0,533 ± 0,109
20:1n-9	0,942 ± 0,091	0,806 ± 0,475	1,141 ± 0,995	2,334 ± 0,091	0,896 ± 0,846*	0,572 ± 0,022	0,672 ± 0,249*
20:3n-9	0,302 ± 0,012	0,765 ± 0,090*	0,513 ± 0,116*	0,635 ± 0,066	0,608 ± 0,132	1,035 ± 0,033	0,618 ± 0,087*
20:3n-6	0,108 ± 0,007	1,519 ± 0,396*	1,009 ± 0,332*	1,222 ± 0,042	0,899 ± 0,318*	1,222 ± 0,030	1,357 ± 0,304*
20:4n-6	2,166 ± 0,109	12,755 ± 2,656*	9,251 ± 3,097*	4,347 ± 0,511	8,240 ± 4,173*	4,220 ± 0,060	16,422 ± 2,357*
20:3n-3	0,000 ± 0,000	0,041 ± 0,076	0,059 ± 0,119	0,097 ± 0,013	0,000 ± 0,000*	0,150 ± 0,015	0,025 ± 0,059*
20:5n-3	0,042 ± 0,013	0,098 ± 0,112	0,166 ± 0,301	0,572 ± 0,038	0,113 ± 0,165*	0,689 ± 0,017	0,138 ± 0,100*
22:0	0,946 ± 0,114	0,978 ± 0,579	1,642 ± 0,591*	0,409 ± 0,018	1,356 ± 0,435*	0,369 ± 0,085	0,492 ± 0,152
22:1n-9	0,144 ± 0,018	1,588 ± 0,595*	2,725 ± 1,570*	0,223 ± 0,024	2,014 ± 1,418*	0,067 ± 0,008	0,664 ± 0,430*
22:2n-6	0,000 ± 0,000	0,000 ± 0,000	0,024 ± 0,067	0,117 ± 0,018	0,000 ± 0,000*	0,074 ± 0,005	0,031 ± 0,045
23:0	0,056 ± 0,013	0,216 ± 0,277	0,239 ± 0,250	0,089 ± 0,015	0,087 ± 0,175	0,027 ± 0,013	0,057 ± 0,053
22:4n-6	0,747 ± 0,103	1,816 ± 0,314*	2,662 ± 1,945*	0,684 ± 0,092	1,545 ± 0,610*	0,278 ± 0,020	3,553 ± 0,446*
22:5n-6	0,164 ± 0,026	0,356 ± 0,110*	0,234 ± 0,189	0,216 ± 0,034	0,431 ± 0,754	0,296 ± 0,027	0,624 ± 0,227*
22:5n-3	1,074 ± 0,121	1,300 ± 0,444	0,855 ± 0,315	1,723 ± 0,069	0,726 ± 0,279*	1,653 ± 0,026	2,376 ± 0,445*
24:0	0,000 ± 0,000	0,557 ± 0,345*	0,809 ± 0,737*	0,073 ± 0,026	0,606 ± 0,292*	0,000 ± 0,000	0,307 ± 0,135*
22:6n-3	1,479 ± 0,077	2,672 ± 1,315	2,852 ± 2,253	2,835 ± 0,093	2,040 ± 1,799	3,481 ± 0,077	3,050 ± 1,187
24:1n-9	1,872 ± 0,190	0,035 ± 0,098*	0,098 ± 0,276*	0,737 ± 0,071	0,064 ± 0,180*	0,139 ± 0,017	0,123 ± 0,149
Ʃ SFA	48,158 ± 1,776	58,067 ± 5,419*	63,738 ± 5,544*	48,229 ± 1,230	67,687 ± 7,719*	47,040 ± 0,881	46,936 ± 4,789*
Ʃ MUFA	40,653 ± 1,636	12,812 ± 1,675*	12,351 ± 2,609*	33,715 ± 1,303	11,846 ± 3,172*	36,304 ± 0,505	17,705 ± 1,311*
Ʃ PUFA	9,621 ± 0,343	28,844 ± 4,890*	23,526 ± 4,114*	16,711 ± 0,464	20,049 ± 5,101*	14,890 ± 0,388	35,118 ± 3,867*
Ʃ trans FA	1,569 ± 0,034	0,276 ± 0,125*	0,385 ± 0,135*	1,345 ± 0,108	0,417 ± 0,172*	1,766 ± 0,074	0,241 ± 0,100*
Ʃ Omega3	2,896 ± 0,153	4,507 ± 1,587	4,533 ± 2,154	5,552 ± 0,145	3,415 ± 1,870	6,104 ± 0,126	5,770 ± 1,552
Ʃ Omega5	0,047 ± 0,028	0,000 ± 0,000*	0,000 ± 0,000*	0,000 ± 0,000	0,000 ± 0,000	0,041 ± 0,009	0,000 ± 0,000*
Ʃ Omega6	6,422 ± 0,208	23,572 ± 4,204*	18,481 ± 4,052*	10,525 ± 0,555	16,026 ± 5,418*	7,751 ± 0,274	28,730 ± 3,304*
Ʃ Omega7	12,709 ± 0,509	2,465 ± 0,376*	2,004 ± 0,477*	10,358 ± 0,511	1,789 ± 0,313*	12,519 ± 0,249	1,806 ± 0,291*
Ʃ Omega9	28,199 ± 1,160	11,112 ± 1,515*	10,861 ± 2,450*	23,992 ± 0,959	10,665 ± 3,083*	24,779 ± 0,333	16,516 ± 1,116*
UI	73,097 ± 2,362	109,691 ± 17,760*	92,754 ± 17,734*	92,332 ± 1,687	78,864 ± 20,728*	92,934 ± 1,835	141,417 ± 15,994*
PI	43,162 ± 1,357	91,565 ± 17,034*	79,091 ± 19,319*	69,931 ± 1,054	65,462 ± 16,533	73,093 ± 1,495	118,882 ± 15,487*

Membrane fatty acid profile of Jurkat, Raji and THP-1 cells compared to the membrane fatty acid profile of human leukocyte subclasses. Data are expressed in weight % of total membrane fatty acids and presented as means ± SD (*n* = 5 for Jurkat,Raji and THP-1; *n* = 8 for CD4^+^, CD8, CD19^+^ and CD14^+^ * Statistically significant difference (*P* < 0.05) from the respective immortalised cell line

The article "Membrane fatty acid heterogeneity of leukocyte classes is altered during in vitro cultivation but can be restored with ad-hoc lipid supplementation" was published in 2015. Journal: Lipids Health Dis.

### Cultured primary lymphocytes have different membrane fatty acid compositions from their primary leukocyte counterparts

The effect of culturing primary human lymphocytes on their membrane fatty acid composition was investigated; results are shown in Table 5. The culture period was 96 h, and cells were cultured either non-stimulated or stimulated with the mitogen PHA. Cultured lymphocytes show an altered membrane fatty acid profile when compared with freshly isolated ones (Table 5). In particular, membranes of cultured lymphocytes were characterized by lower proportions of oleic acid, monounsaturated fatty acids and PUFAs. Conversely membranes of freshly isolated lymphocytes had higher proportions of palmitic, stearic and total saturated fatty acids. Stimulating the lymphocytes with the mitogen PHA had only modest effects on membrane fatty acid composition beyond those seen with culture itself, except that the proportion of arachidonic acid was significantly lower after stimulation (Table 5).

**Table 5:** Membrane fatty acid profile comparison between freshly isolated and primary lymphocytes

	Freshly isolated lymphocytes	Primary lymphocytes 96 h - non stimulated	Primary lymphocytes 96 h - PHA stimulated
14:0	0,426 ± 0,024^ab^	0,678 ± 0,079^ac^	0,801 ± 0,062^bc^
15:0	0,196 ± 0,012^ab^	0,273 ± 0,058^a^	0,300 ± 0,055^b^
16:0	22,772 ± 1,171^ab^	28,499 ± 1,267^ac^	31,641 ± 1,304^bc^
t16:1n-7	0,261 ± 0,011	0,268 ± 0,028	0,316 ± 0,052
16:1n-7	0,281 ± 0,011^ab^	0,180 ± 0,011^ac^	0,233 ± 0,014^bc^
17:0	0,448 ± 0,025^ab^	0,717 ± 0,173^a^	0,770 ± 0,145^b^
17:1	0,065 ± 0,017^ab^	0,000 ± 0,000^a^	0,000 ± 0,000^b^
18:0	24,839 ± 1,710^ab^	30,630 ± 1,045^a^	32,467 ± 1,992^b^
t18:1n-9	0,000 ± 0,000	0,025 ± 0,049	0,041 ± 0,058
18:1n-9	15,653 ± 0,557^ab^	9,182 ± 0,084^a^	9,310 ± 0,882^b^
18:1n-7	2,076 ± 0,119^ab^	1,222 ± 0,027^a^	1,307 ± 0,209^b^
18:2n-6	6,512 ± 0,250^ab^	3,330 ± 0,085^a^	3,310 ± 0,231^b^
18:3n-6	0,077 ± 0,013^ab^	0,096 ± 0,006^ac^	0,130 ± 0,025^bc^
18:3n-3	0,117 ± 0,025^a^	0,254 ± 0,127^a^	0,255 ± 0,122
20:0	0,604 ± 0,040^ab^	1,106 ± 0,167^a^	1,153 ± 0,141^b^
20:1n-9	0,908 ± 0,073^ab^	0,517 ± 0,013^a^	0,524 ± 0,067^b^
20:3n-9	0,634 ± 0,036^ab^	0,333 ± 0,039^a^	0,402 ± 0,123^b^
20:3n-6	1,522 ± 0,083^ab^	1,137 ± 0,089^a^	1,024 ± 0,177^b^
20:4n-6	15,726 ± 0,900^ab^	12,940 ± 1,163^ac^	8,644 ± 1,592^bc^
20:5n-3	0,182 ± 0,018	0,227 ± 0,017^c^	0,170 ± 0,032^c^
22:0	0,301 ± 0,064^ab^	1,018 ± 0,371^a^	1,070 ± 0,441^b^
22:1n-9	0,082 ± 0,011^ab^	0,108 ± 0,015^a^	0,113 ± 0,023^b^
22:2n-6	0,080 ± 0,009^b^	0,117 ± 0,019^c^	0,000 ± 0,000^bc^
23:0	0,000 ± 0,000^ab^	0,167 ± 0,031^a^	0,185 ± 0,057^b^
22:4n-6	2,370 ± 0,104^b^	2,532 ± 0,294^c^	1,676 ± 0,303^bc^
22:5n-6	0,469 ± 0,075	0,686 ± 0,367	1,488 ± 2,231
22:5n-3	1,526 ± 0,076^ab^	1,558 ± 0,057^ac^	1,063 ± 0,174^bc^
22:6n-3	1,872 ± 0,094	2,197 ± 0,102^c^	1,606 ± 0,222^c^
Ʃ SFA	49,588 ± 1,998^ab^	63,089 ± 1,234^ac^	68,386 ± 2,794^bc^
Ʃ MUFA	19,065 ± 0,742^ab^	11,209 ± 0,068^a^	11,488 ± 1,106^b^
Ʃ PUFA	31,086 ± 1,268^ab^	25,409 ± 1,258^ac^	19,769 ± 2,124^bc^
Ʃ trans FA	0,261 ± 0,011	0,292 ± 0,072	0,357 ± 0,097
Ʃ Omega3	3,697 ± 0,187^b^	4,236 ± 0,133^c^	3,094 ± 0,342^bc^
Ʃ Omega5	0,000 ± 0,000	0,000 ± 0,000	0,000 ± 0,000
Ʃ Omega6	26,756 ± 1,112^ab^	20,839 ± 1,209^ac^	16,272 ± 1,925^bc^
Ʃ Omega7	2,422 ± 0,129^ab^	1,402 ± 0,018^a^	1,540 ± 0,220^b^
Ʃ Omega9	17,276 ± 0,657^ab^	10,141 ± 0,069^a^	10,350 ± 0,928^b^
UI	124,585 ± 5,279^ab^	101,606 ± 4,870^ac^	80,302 ± 9,028^bc^
PI	98,379 ± 3,877^ab^	88,712 ± 4,192^a^	69,943 ± 11,107^b^

Membrane fatty acid profile of freshly isolated lymphocytes compared to the membrane fatty acid profile of primary lymphocytes isolated, non-stimulated/PHA-stimulated and cultivated in vitro for 96 h. Data are expressed in weight % of total membrane fatty acids and presented as means ± SD (*n* = 5 for all). ^a, b, c^ Statistically significant difference (*P* < 0,05) as follows: ^a^ Freshly vs Non stimulated, ^b^ Freshly vs PHA-Stimulated, ^c^ Non stimulated vs PHA-Stimulated

The article "Membrane fatty acid heterogeneity of leukocyte classes is altered during in vitro cultivation but can be restored with ad-hoc lipid supplementation" was published in 2015. Journal: Lipids Health Dis.

### Refeed® supplementation realigns Jurkat membrane fatty acid composition to that of primary human CD4^+^ lymphocytes

Jurkat cells were cultured in the traditional medium (RPMI + 10 % FBS) supplemented with specific Refeed® supplements, which are completely defined combinations of lipids and lipophilic antioxidants (see Methods). Culture with Refeed® WT was able to modify and maintain over time the membrane fatty acid profile of Jurkat cells to one that better matched that of primary CD4^+^ lymphocytes from healthy individuals (Table 6). In particular, linoleic and arachidonic acid proportions did not differ from proportions seen in the fresh CD4^+^ cells (Table 6). None of the ten summary parameters was different between primary CD4^+^ lymphocytes and Refeed® WT supplemented Jurkat cells, while they were all different between traditionally cultured Jurkat cells and primary CD4^+^ cells (Table 6). Therefore, the membrane network of Refeed® WT supplemented Jurkat cells mimics that of freshly isolated primary CD4^+^ lymphocytes in its fatty acid composition and so most likely in its biophysical and functional properties.

**Table 6:** Effect of lipid supplementation on membrane fatty acid profile of Jurkat cells

	CD4+	Jurkat	Jurkat + Refeed WT
12:0	0,000 ± 0,000	0,056 ± 0,011*	0,000 ± 0,000
14:0	0,635 ± 0,190	2,062 ± 0,085*	0,829 ± 0,155
14:1n-5	0,000 ± 0,000	0,047 ± 0,028*	0,000 ± 0,000
15:0	0,256 ± 0,150	0,194 ± 0,012*	0,172 ± 0,094
16:0	27,156 ± 1,864	25,776 ± 2,014	21,420 ± 2,863*
t16:1n-7	0,265 ± 0,133	0,834 ± 0,036*	0,236 ± 0,084
16:1n-7	0,257 ± 0,140	7,188 ± 0,407*	0,422 ± 0,229
17:0	0,696 ± 0,169	0,411 ± 0,050*	0,650 ± 0,299
18:0	26,877 ± 3,827	18,049 ± 0,606*	29,737 ± 2,063
t18:1n-9	0,012 ± 0,033	0,735 ± 0,033*	0,089 ± 0,142
18:1n-9	7,919 ± 1,053	24,938 ± 1,156*	11,018 ± 1,526*
18:1n-7	2,208 ± 0,375	5,521 ± 0,356*	2,104 ± 0,851
18:2n-6	6,946 ± 1,323	3,144 ± 0,210*	7,446 ± 1,034
18:3n-6	0,179 ± 0,118	0,094 ± 0,017	0,235 ± 0,132
18:3n-3	0,396 ± 0,319	0,302 ± 0,036	0,296 ± 0,101
20:0	0,697 ± 0,241	0,608 ± 0,045	0,753 ± 0,377
20:1n-9	0,806 ± 0,475	0,942 ± 0,091	0,634 ± 0,231
20:3n-9	0,765 ± 0,090	0,302 ± 0,012*	0,757 ± 0,091
20:3n-6	1,519 ± 0,396	0,108 ± 0,007*	2,110 ± 0,592
20:4n-6	12,755 ± 2,656	2,166 ± 0,109*	12,296 ± 1,326
20:3n-3	0,041 ± 0,076	0,000 ± 0,000	0,004 ± 0,009
20:5n-3	0,098 ± 0,112	0,042 ± 0,013	0,133 ± 0,114
22:0	0,978 ± 0,579	0,946 ± 0,114	0,448 ± 0,168*
22:1n-9	1,588 ± 0,595	0,144 ± 0,018*	0,081 ± 0,021*
22:2n-6	0,000 ± 0,000	0,000 ± 0,000	0,000 ± 0,000
23:0	0,216 ± 0,277	0,056 ± 0,013	0,258 ± 0,197
22:4n-6	1,816 ± 0,314	0,747 ± 0,103*	4,457 ± 0,385*
22:5n-6	0,356 ± 0,110	0,164 ± 0,026*	0,262 ± 0,068
22:5n-3	1,300 ± 0,444	1,074 ± 0,121	0,670 ± 0,072*
24:0	0,557 ± 0,345	0,000 ± 0,000*	0,069 ± 0,012*
22:6n-3	2,672 ± 1,315	1,479 ± 0,077	2,413 ± 1,232
24:1n-9	0,035 ± 0,098	1,872 ± 0,190*	0,000 ± 0,000
Ʃ SFA	58,067 ± 5,419	48,158 ± 1,776*	54,337 ± 2,323
Ʃ MUFA	12,812 ± 1,675	40,653 ± 1,636*	14,259 ± 1,005
Ʃ PUFA	28,844 ± 4,890	9,621 ± 0,343*	31,078 ± 2,759
Ʃ trans FA	0,276 ± 0,125	1,569 ± 0,034*	0,326 ± 0,180
Ʃ Omega3	4,507 ± 1,587	2,896 ± 0,153	3,516 ± 1,119
Ʃ Omega5	0,000 ± 0,000	0,047 ± 0,028*	0,000 ± 0,000
Ʃ Omega6	23,572 ± 4,204	6,422 ± 0,208*	26,806 ± 2,474
Ʃ Omega7	2,465 ± 0,376	12,709 ± 0,509*	2,526 ± 0,911
Ʃ Omega9	11,112 ± 1,515	28,199 ± 1,160*	12,489 ± 1,447
UI	109,691 ± 17,760	73,097 ± 2,362*	126,496 ± 10,755
PI	91,565 ± 17,034	43,162 ± 1,357*	93,767 ± 11,347

Membrane fatty acid profile of fresh CD4^+^ human T lymphocytes compared to the membrane fatty acid profile of traditionally cultured Jurkat cells and the membrane fatty acid profile of Refeed® WT supplemented Jurkat cells. Data are expressed in weight % of total membrane fatty acids and presented as means ± SD (*n* = 8 for CD4^+^, *n* = 5 for traditionally cultured Jurkat cells, *n* = 5 for Refeed® WT supplemented Jurkat cells). * Statistically significant difference (*P* < 0.05)

Jurkat cells were also incubated with Refeed® CVD and with Refeed® O3+ and were characterized by a fatty acid composition very consistent over culture passages. Figure 1 summarises the membrane fatty acid composition data for these cells as well as for fresh primary CD4^+^ T lymphocytes, Jurkat cells cultured with standard medium and Jurkat cells cultured with Refeed® WT. Incubation of Jurkat cells with Refeed® WT, Refeed® CVD or Refeed® O3+ resulted in Jurkat cells with proportions of saturated, monounsaturated, polyunsaturated, n-6 polyunsaturated and arachidonic acids that were similar to those seen in fresh primary CD4^+^ T lymphocytes and quite different from those seen normally in cultured Jurkat cells (Fig. 1). Incubation with Refeed® CVD resulted in Jurkat cells with an elevated proportion of trans fatty acids and a decreased proportion of n-3 PUFAs including docosahexaenoic acid (Fig. 1). Conversely incubation with Refeed® O3+ resulted in Jurkat cells with lower proportions of arachidonic acid and n-6 PUFAs and higher proportions of docosahexaenoic acid and n-3 PUFAs (Fig. 1).

The article "Membrane fatty acid heterogeneity of leukocyte classes is altered during in vitro cultivation but can be restored with ad-hoc lipid supplementation" was published in 2015. Journal: Lipids Health Dis.

**Fig. 1:** Comparison of main fatty acid membrane parameters of in-vivo and in-vitro leukocytes. The main fatty acid parameters characterizing the membrane fatty acid profile of CD4^+^ (primary fresh uncultured CD4^+^ T lymphocytes), JC (Jurkat cells cultured under traditional conditions), WT (Jurkat cells supplemented with Refeed® WT), CVD (Jurkat cells supplemented with Refeed® CVD), O3+ (Jurkat cells supplemented with Refeed® O3+). Data are expressed as % of controls (CD4+) and presented as means ± SD (*n* = 8 for CD4+, *n* = 5 for JC, WT, CVD, O3+). * Statistically significant difference (*P* < 0.05)

## Discussion

Leucocytes are composed of different classes of cells, including CD4^+^ T-lymphocytes, CD8^+^ T-lymphocytes, B lymphocytes and monocytes; each cell class has specific functions within the immune system. Numerous studies have noted the importance of the membrane network within specific leukocyte classes, highlighting how the functional diversity of these cells is extremely refined and very often linked to changes in the membrane fatty acid profile, with consequences that affect membrane biophysical properties. Nevertheless, the current literature lacks a systematic comparison between the main leukocyte classes concerning their membrane fatty acid composition. Here we identified marked differences in membrane fatty acid composition among the four leukocyte subclasses studied. In particular, monocytes had quite a different membrane fatty acid profile from lymphocytes. Furthermore, it is interesting that even closely related cells such as CD4^+^ and CD8^+^ T-lymphocytes are different from one another. The membrane composition of the leukocytes was summarized according to particular characteristics (e.g. UI) that might be related to function, at least at the level of the membrane. Indeed membrane-mediated events are able to be modulated by changing the fatty acid composition of the membrane, as clearly demonstrated for phagocytosis [24, 29]. The four leukocyte classes studied differed according to the summary characteristics, again with monocytes being quite different from lymphocytes. Although there are many reports of the fatty acid composition of specific leukocyte classes such as neutrophils [30–33] and mononuclear cells [24, 34–37] very few studies have made comparisons between different leukocyte classes before. Perhaps the most detailed previous example is Gibney and Hunter [38] who compared the fatty acid composition of human blood neutrophils, T-lymphocytes, B-lymphocytes and monocytes. They found differences amongst these four cell types, in general agreement with the current study.

The article "Membrane fatty acid heterogeneity of leukocyte classes is altered during in vitro cultivation but can be restored with ad-hoc lipid supplementation" was published in 2015. Journal: Lipids Health Dis.

The second key finding of the current study is that the membrane fatty acid composition is markedly different between fresh primary human leukocytes and comparator immortalized cell lines that are commonly used in research. This would suggest that the cell lines as currently cultured may not represent an optimal situation with which to make conclusions about in vivo or physiological processes. All three immortalized cell lines were characterised by a significant deficit of PUFAs and n-6 PUFAs, in particular of arachidonic acid, a biologically important fatty acid from which over one hundred bioactive lipids can be formed. The membrane fatty acid profile of all three cell lines was very consistent over several in vitro passages (data not shown). An interesting observation was that the membrane fatty acid profiles of the three cell lines were rather different from one another, even though the cells were grown in exactly the same culture medium and with the same batch of FBS. This observation shows the cells are able to control their membrane fatty acid composition suggesting metabolic and/or genetic mechanisms as being responsible. Nevertheless it is known that adding specific fatty acids to the culture medium can modify the membrane fatty acid composition of cultured primary leukocytes [29, 39] and cultured leukocytic cell lines [40, 41]. Indeed in the current study it was observed that adding mixtures of fatty acids to Jurkat cells resulted in an altered membrane fatty acid composition. By tailoring the fatty acid mixture added to the medium, Jurkat cells could be produced that had a membrane fatty acid profile more closely resembling that of fresh primary human T-lymphocytes. Other fatty acid mixtures produced Jurkat cells enriched in n-3 PUFAs, perhaps mimicking fish oil supplementation, or enriched in trans fatty acids. These modifications may enable the development of innovative experimental models that can mimic specific physiological or pathological conditions, or even the membrane conditions of specific human populations and/or deriving from specific dietary intakes. This would represent a significant advance in experimental capabilities.

The article "Membrane fatty acid heterogeneity of leukocyte classes is altered during in vitro cultivation but can be restored with ad-hoc lipid supplementation" was published in 2015. Journal: Lipids Health Dis.

The final key finding of the current study is that after four days of cultivation in vitro, primary lymphocytes showed membrane fatty acid profiles which were very different from the original freshly prepared cells, and the changes were in line with what was already observed for immortalized cells. In particular, there was a decrease of PUFA, of n-6 PUFA and of arachidonic acid, and so likely a decrease in membrane fluidity. Membranes of lymphocytes cultured for 96 h showed a 50 % lower content of linoleic acid and an 18 % lower content of arachidonic acid compared with fresh cells. The decreased content of arachidonic acid was exaggerated by mitogen stimulation (45 % lower content than fresh cells). Anel et al. [42] reported effects of quiescent and mitogen-stimulated culture for 72 h on the fatty acid composition of human mononuclear cells and purified T-lymphocytes. They identified that culture resulted in lower contents of both linoleic and arachidonic acid (30 % and 19 %, respectively) in purified T-lymphocytes, changes that were exaggerated by mitogenic stimulation. Likewise, Calder et al. [39] reported that culture of mitogen-stimulated rat lymphocytes for 48 h resulted in lower contents of linoleic and arachidonic acids (45 % and 25 % lower respectively) than seen in freshly prepared cells. These changes in fatty acid composition were associated with changes in membrane fluidity and T-lymphocyte function [39, 42], establishing a clear link between membrane fatty acid content, membrane physical properties and leukocyte function [25]. Thus, it is likely that the differences in leukocyte membrane fatty acid content reported in the current study have a functional significance.

The findings of the current study suggest that the classical method of in vitro cultivation of leukocytes is not optimal, when the membrane, its fatty acid content and its biophysical properties are taken into consideration. It is evident that comparison of fresh primary cells with those produced in vitro and the development of customized in vitro supplementation to mimic different nutritional, physiological and pathological contexts should become more routine practice when using these cell lines. If not, it seems highly likely that the large in vivo versus in vitro difference is likely to lead to highly biased experimental data.

The article "Membrane fatty acid heterogeneity of leukocyte classes is altered during in vitro cultivation but can be restored with ad-hoc lipid supplementation" was published in 2015. Journal: Lipids Health Dis.

The use of customized lipid supplementation may represent an important tool to evolve in vitro experimental models. By changing the quality and quantity of the components of the supplement in order to act on specific pathways of synthesis and control of the lipid metabolism, it is possible to produce cell membranes with a very different fatty acid profile, perhaps representing different in vivo nutritional exposures, and even typical of specific physiological and pathological conditions.

## Conclusions

The present study shows that the various classes of leukocytes have a specific membrane fatty acid profile in vivo that is unlike that of other leukocytes, and which makes the membrane properties of different cell types different and probably better aligned with their function. However, the specific characteristics of the membrane are completely lost during the in vitro cultivation of primary leukocytes. Furthermore primary leukocytes have very different membrane fatty acid compositions from commonly studied comparator immortalized cell lines. This in vivo versus in vitro membrane dichotomy makes the currently used in vitro experimental models inadequate. Culture of primary lymphocytes results in changes in fatty acid composition. Addition of specific mixtures of fatty acids to the culture medium can be used to modify the fatty acid composition of immortalized cell lines (in this case Jurkat cells) to much better resemble that of freshly prepared human blood lymphocytes. Such customised lipid preparations can be used to improve in vitro research with immortalised leukocytic cell lines. The development of customised lipid supplements can greatly aid the development of innovative experimental models that can mimic specific physiological or pathological conditions, or even the membrane conditions of specific human populations and/or deriving from specific dietary intakes, thus expanding the quality of in vitro studies and guaranteeing the availability of better quality experimental data for scientific research and for the development of new drugs and innovative therapies.

## Abbreviations

ATCC: American Type Culture Collection
FAMEs: fatty acid methyl esters
FBS: fetal bovine serum
MUFA: mono-unsaturated fatty acids
PBMCs: peripheral blood mononuclear cells
PI: Peroxidability Index
PHA: phytohaemagglutinin
PUFA: poly-unsaturated fatty acids
SFA: saturated fatty acids
UFA: unsaturated fatty acids
UI: Unsaturation Index
